This article has been retracted.

# Screening and functional prediction of differentially expressed genes in walnut endocarp during hardening period based on deep neural network under agricultural internet of things

**DOI:** 10.1371/journal.pone.0263755

**Published:** 2022-02-24

**Authors:** Zhongzhong Guo, Shangqi Yu, Jiazhi Fu, Kai Ma, Rui Zhang

**Affiliations:** 1 College of Life Science, Tarim University, Alar, Xinjiang, China; 2 Key Laboratory of Biological Resource Protection and Utilization of Tarim Basin Xinjiang Production and Construction Group, Alar, Xinjiang, China; 3 The National and Local Joint Engineering Laboratory of High Efficiency and Superior-Quality Cultivation and Fruit Deep Processing Technology of Characteristic Fruit Trees in South Xinjiang, Alar, Xinjiang, China; 4 College of Horticulture and Forestry Sciences, Tarim University, Alar, Xinjiang, China; 5 Research Institute of Horticultural Crops, Xinjiang Academy of Agricultural Sciences, Urumqi, China; Ministry of Natural Resources North Sea Bureau, CHINA

## Abstract

The deep neural network is used to establish a neural network model to solve the problems of low accuracy and poor accuracy of traditional algorithms in screening differentially expressed genes and function prediction during the walnut endocarp hardening stage. The paper walnut is used as the research object to analyze the biological information of paper walnut. The changes of lignin deposition during endocarp hardening from 50 days to 90 days are observed by microscope. Then, the Convolutional Neural Network (CNN) and Long and Short-term Memory (LSTM) network model are adopted to construct an expression gene screening and function prediction model. Then, the transcriptome and proteome sequencing and biological information of walnut endocarp samples at 50, 57, 78, and 90 days after flowering are analyzed and taken as the training data set of the CNN + LSTM model. The experimental results demonstrate that the endocarp of paper walnut began to harden at 57 days, and the endocarp tissue on the hardened inner side also began to stain. This indicates that the endocarp hardened laterally from outside to inside. The screening and prediction results show that the CNN + LSTM model’s highest accuracy can reach 0.9264. The Accuracy, Precision, Recall, and F1-score of the CNN + LSTM model are better than the traditional machine learning algorithm. Moreover, the Receiver Operating Curve (ROC) area enclosed by the CNN + LSTM model and coordinate axis is the largest, and the Area Under Curve (AUC) value is 0.9796. The comparison of ROC and AUC proves that the CNN + LSTM model is better than the traditional algorithm for screening differentially expressed genes and function prediction in the walnut endocarp hardening stage. Using deep learning to predict expressed genes’ function accurately can reduce the breeding cost and significantly improve the yield and quality of crops. This research provides scientific guidance for the scientific breeding of paper walnut.

## Introduction

Biological data is growing exponentially with the rapid development of life science and computer science. This growth dramatically enriches the data resources of bioinformatics in terms of quality and quantity and provides a data basis for solving the mystery of life. The prediction and functional screening of crops’ expressed genes can be used for environmental detection, prevention, control, drug screening, and complex disease diagnosis, especially in selecting optimal product breeding. The screening and functional prediction of differentially expressed genes can significantly improve the yield and quality of crops. Walnuts, as a widely distributed economic crop in China [1], are mainly distributed in Xinjiang and other places. Walnuts can be eaten and oiled with high economic value and nutritional value. Moreover, the walnut shell has high calorific value [2, 3], so it can be used as fuel. Walnut kernels are rich in nutrients such as vitamin B, melatonin, and antioxidants, which are beneficial to improving memory and ameliorating neurasthenia. The quality of walnut kernels and the thickness of walnut shell are the primary indicators to measure the quality of walnuts. Therefore, cultivating thin-shell walnuts is also one of the goals of walnut breeding [4, 5].

At present, walnut planting, walnut high yield, and walnut quality are the principal contents and directions of research. The thin-shell walnuts in the Aksu area of Xinjiang have adequate quality and extensive market prospects. The genotypes of early-maturing and late-maturing walnuts were studied by Wang et al. [6]. The authors analyzed the growth process, photosynthetic ability, and non-photosynthetic ability (carbohydrate content, chloride ion distribution, reactive oxygen species (ROS) accumulation, and osmotic adjustment under water stress, salinity, and their combination) of the two walnuts. They found that compared with early-maturing walnuts, late-maturing walnuts showed higher total biomass and net photosynthetic rate, higher antioxidant enzyme activity, higher osmotic adjustment and lower reactive oxygen species accumulation under stress conditions. Moreover, late-maturing walnuts had better stress resistance under water stress and salt stress. Khadivi et al. [7] investigated how to screen out the spring frost resistant genotypes with high grain quality and quantity value from mature seedlings. Their research results showed that 67 mature seedling genotypes bloomed late and were not exposed to frost, and the genotypes showed significant differences in all measured fruit traits. The nut weight ranged from 7.53 g to 16.91 g, while the grain weight ranged from 3.17 g to 8.23 g, and the percentage of grains ranged from 39.44% to 68.14%. Walters et al. [8] reviewed the latest research results on the composition, classification, extraction methods, in vivo functions, and clinical functions of different parts of walnuts. The authors summarized those foods rich in walnuts had significant improvement on chronic diseases, and the mechanism was that different components of walnuts synergistically or independently played antioxidant and anti-inflammatory effects. These studies have opened up new ways to enhance the impact of walnuts on human health and accelerated the development and utilization of walnuts in functional foods. Li et al. [9] proposed a new prediction method based on deep learning technology. This method adopted the trained Convolutional Neural Network (CNN) for prediction and took the coding vector of gene sequence as input without manually extracting sample features. Through experiments, they found that the main performance indexes of the prediction model, including the Matthews correlation coefficient, were more sensitive than the traditional machine learning methods. Wang et al. put forward a gene expression prediction model based on the Long and Short-term Memory (LSTM) neural network. The model captured the nonlinear features affecting gene expression and used the learned features to predict the target gene. The comparison and analysis of experimental errors and the fitting effects of different prediction models proved that the LSTM neural network model could achieve lower error and better fitting results [10].

Based on the above research, this paper takes paper walnut as the research object. Firstly, the changes of lignin deposition of paper walnut during endocarp hardening from 50 days to 90 days in the growth period are observed to analyze the biological information of walnut. Then, the expression gene screening and the prediction model is established by using CNN and LSTM. In the experiment, the CNN + LSTM model is used to comprehensively analyze all the genes expressed in the endocarp hardening stage of paper walnut. The gene screening and function prediction model established here is compared with the prediction results of traditional models. The research reported here provides scientific guidance for the breeding and planting of paper walnut.

## Research materials and methods

### Experimental materials

The materials used in this experiment are thin-shell walnuts [11, 12] produced in Aksu, Xinjiang. The flesh of thin-shell walnuts begins to develop 50 days after the flowering stage, and the flesh changes from growth stage to hardening stage that lasts for 30 days. According to the growth and development law of thin-shell walnuts, samples are randomly collected in 50 days, 57 days, 78 days, and 90 days after the full-bloom stage from different parts of the tree. Fifty samples are collected each time, and then the samples are processed under low temperature conditions. Specifically, the green skin outside the walnut, fruit skin, and kernel skin are removed, and then the flesh part is ground to powder and mixed thoroughly with a stirring device, and then the power is frozen with liquid nitrogen and stored in a thermostat at 80°C below zero.

### Sample processing procedure

(1) Dyeing of thin-shell walnut flesh [13, 14]: the mixed solution A with a volume ratio of 1: 1 is prepared by anhydrous ethanol and concentrated hydrochloric acid. Then, phloroglucinol is dissolved by the solution A to prepare the mixed solution B containing 3% phloroglucinol solution. The mixed solution B is experimental dye liquor. Finally, the thin-shell nut flesh is placed in the dye liquor for 5 to 6 minutes until the lignin is dyed pink. Then, the sample is observed and photographed under the microscope. The solution after standing is light yellow, and the solution can be sealed preserved in the brown reagent bottle for about 15 days.

(2) RNA extraction from the fruit of thin-shell walnuts [15]: RNA is extracted from the fruit by a RNA extractor, and each sample is subjected to multiple RNA extraction. According to the test results, the samples with the requirements of RNA sequencing are mixed and used as the final test samples.

### CNN and LSTM

In recent years, as a subset of artificial intelligence and machine learning, the deep learning algorithm greatly simplifies the workflow of machine learning. Deep learning is a concept proposed by American scholars in the second half of the 20th century. Its initial purpose is to explore the degree of learning engagement and mastery of knowledge of learners [16, 17]. In the learning process, different learners may adopt different strategies to achieve the purpose of knowledge acquisition. Learning methods can be simply divided into deep learning and shallow learning. Deep learning means that learners think, understand, and raise their own problems in the learning process. Shallow learners do not pay attention to the understanding of knowledge, but acquire knowledge through passive memory. Obviously, deep learning is better than shallow learning. Fig 1 reveals the further comparison between deep learning and shallow learning [18].

**Fig 1:** Comparison between deep learning and shallow learning.

At present, there is no unified definition of deep learning. However, by referring to relevant literature, most scholars define deep learning from the following four aspects [19, 20] as shown in Fig 2.

**Fig 2:** Definition to deep learning.

The most significant feature of deep learning is having multiple hidden layers [21]. Using the function transformation to transfer the input data to the first layer, the output can be expressed as Eq (1).


$$R_{1}=f(W_{1}*X+B_{1})$$ (1)

In Eq (1), *R*_*1*_ refers to the output matrix of the first hidden layer, *f* signifies the activation function, *W*_*1*_ denotes the weight matrix, and *B*_*1*_ represents the threshold matrix. The output of the *m*-th hidden layer can be written as Eq (2) [22].


$$R_{m}=f(W_{m}\cdot R_{m-1}+B_{m})$$ (2)

Similarly, the final output is:

$$y_{k}=g(W_{n+1}\cdot R_{n}+B_{n+1})$$ (3)

where *g* denotes the classification function of the output layer.

The deep learning methods used here primarily include CNN, Recurrent Neural Network (RNN), and LSTM network.

(1) CNN

CNN is one of the most representative algorithms among deep learning [23], and it is a pre-feedback network structure that supervises learning ability. Convolution operation refers to the identification of input data characteristics through convolution check. The convolution kernel that inputs data and the grid structure are relatively regular, which can be stored in the form of multidimensional arrays. The size of convolution kernels is not clearly defined, but it cannot exceed the size of input data. Convolution operation is especially effective for some types of data, which uses invariant data attributes, such as spatial local attributes and translation invariance, to analyze input data and identify the features of the input data by convolution checking. In addition, CNN uses the same convolution kernel in the process of data input, so it requires fewer parameters for data operation and analysis than traditional neural networks, which makes the whole analysis process extremely simple. Therefore, this data processing method is also called data parameter sharing. Sequence-based parameters can be seen as text data containing vast quantities of information. CNN can achieve excellent effects on gene screening and functional prediction. Fig 3 illustrates the structure of CNN [24, 25]. Fig 4 displays the composition of CNN [26].

**Fig 3:** Structure of CNN.

**Fig 4:** Composition of CNN.

Through Fig 3, a CNN mainly consists of the input layer, the hidden layer, and the output layer, and the hidden layer includes the convolution layer, the pooling layer, and the fully connected layer. The operation of convolution operators on real values can theoretically be expressed by Eq (4).


y(z)=(x*w)(z)=∫x(t)w(z−t)dt (4)

In Eq (4), *x* (*t*) represents the input value on the *t* position, and *w* refers to the convolution kernel. Eq (4) can be regarded as the weighted average of *w* in the whole neighborhood of *x*. If the input data are multi-dimensional, the above function can be replaced by multivariate. If the input data are discrete, the above operation can be replaced by summation. For example, the convolution operation using the two-dimensional kernel *w* on the two-dimensional image *x* can be presented as Eq (5).


$$y(m,n)=(x*w)(m,n)=\sum_{i,j}x(i,j)w(m-i,n-j)$$ (5)

Eq (5) represents the pixel value of coordinate (*m*, *j*). The center of convolution kernel is placed on the corresponding pixel position, and the sum of the corresponding pixel product and the overlapping parameters is calculated. Finally, the output at position (*m*, *n*) is obtained. The above process is the basis of convolution operation in CNN. Through this operation, different features of the input data can be extracted.

(2) LSTM

LSTM is a kind of RNN, which can handle time series dependent events effectively [27, 28]. Each LSTM unit contains an input gate, an output gate, and several forgetting gates. Among them, the main function of the input gate is to control the input data of the model, and the main function of the output gate is to control the output of the model to the calculation results. Besides, the forgetting gate is mainly responsible for calculating the forgetting degree of the memory module at the previous moment. Fig 2 signifies the structure of the LSTM network. Eq (6) indicates the forgetting gate *f*_*t*_ of the LTSM network.


$$f_{t}=\sigma (W_{f}\cdot [h_{t-1},x_{t}]+b_{f}$$ (6)

The input gate *i*_*t*_ can be written as Eq (7). The forgetting gate controls the forgetting degree of each input information, and the input gate controls the degree of each data information newly written into long-term information.


$$i_{t}=\sigma (W_{i}\cdot [h_{t-1},x_{t}]+b_{i}$$ (7)

$$C=\tanh(W_{c}\cdot [h_{t-1},x_{t}]+b_{c}$$ (8)

$$C_{t}=f_{t}\times C_{t-1}+i_{t}\times C$$ (9)

The activation function selected by the forgetting gate *f*_*t*_ and the input gate *i*_*t*_ is the Sigmoid function. The function value of the Sigmoid function is between 0 and 1, and the range of the activation function tanh function is between −1 and 1. Denote *C*_*t*-*1*_ as the state of a neuron at time *t*-*1*, and *C*_*t*_ as the state of a neuron at time *t*.


$$h_{t}=o_{t}\times \tanh(C_{t})$$ (10)

$$o_{t}=\sigma (w_{o}\cdot [h_{t-1},x_{t}]+b_{o}$$ (11)

In Eqs (10) and (11), *o*_*t*_ denotes the output gate that controls the output of information, and *h*_*t*_ represents the output of the *t*th step. Fig 5 shows the structure of the LSTM network.

**Fig 5:** Schematic diagram of LSTM network structure.

(3) Selection of the activation function

In the neural network structure, the output value of the upper layer is the input value of the next layer, and the output node of the upper layer is the input node of the next layer. The activation function is the functional relationship between these nodes. The paramount procedure of constructing a neural network is the selection of activation function. The appropriate activation function can significantly improve the convergence speed and simulation accuracy of the neural network model. Besides, the activation function can introduce nonlinear characteristics into the neural network to strengthen the network. There are three activation functions used for neural networks.

(1) Sigmoid function:

$$Sigmoid(x)=\frac{1}{1+e^{-x}}$$ (12)

(2) Tanh function:

$$Tanh(x)=\frac{sinh(x)}{cosh(x)}=\frac{1‐e^{‐2x}}{1+e^{‐2x}}=‐1+2Sigmoid(x)=‐1+\frac{2}{1+e^{‐2x}}$$ (13)

(3) ReLU function:

$$Relu(x)=max(0,x)=\{\begin{array}{l} 0,otherwise\\ x,ifx,0 \end{array}$$ (14)

Fig 6 provides the curves of three activation functions.

**Fig 6:** Curves of three activation functions.

Three functions have their own advantages and disadvantages. Among them, the ReLU function and Sigmoid function are the most commonly used activation functions. The convergence speed of ReLU function is 6 times faster than that of Sigmoid function, but the fault tolerance rate is low. If the learning rate is improper, it will lead to a gradient of 0. Here, Sigmoid function and ReLU function are selected as activation functions for the model.

## Screening and function prediction model of DEGs based on deep learning

### Data acquisition and pre-processing

(1) Data acquisition.

According to the above experimental design, transcriptome sequencing, proteome sequencing and biological information analysis are performed on the endocarp samples of walnuts during the four periods of 50 days, 57 days, 78 days and 90 days after full bloom. There is a total of 77,570 mRNA and 6,776 protein expression data used as the initial data of training the CNN + LSTM model based on deep learning. Then, base substitution and complement are used to process the data [29], and all the gene sequences are complemented to 25nt.

(2) Data pre-processing.

The data set is obtained through data acquisition, and the data need to be pre-processed to obtain the input data of the neural network model. The computer binary is used for reference. The data combination form of 0 and 1 is the most easily recognized for computers. Therefore, four bases, adenine (A), thymine (T), guanine (G), and cytosine (C), can be represented by four-bit one-hot encoding. According to the above base substitution, T is replaced by U. The data are pre-processed by this method. For instance, Fig 7 provides the principle of encoding the RNA sequence {UUGAAGAGGACUUGGA}.

**Fig 7:** Four-bit one-hot encoding of the RNA sequence.

According to Fig 7, by encoding the gene sequence {UUGAAGGACUUGGA}, it is expressed as a two-dimensional vector of 16 × 4, so that the gene data can be processed into data that can be input into the neural network model.

(3) Setting of data labels.

After coding the data, it is essential to set data labels by marking “1” as the positive target gene data of RNA and marking “0” as the negative target gene data of RNA.

### Implementation of the network model

The screening and functional prediction of DEGs in the endocarp of thin-shell walnuts can be regarded as a data classification problem. In this experiment, CNN and LSTM algorithms are combined to screen genes and predict functions. The LSTM model can predict functions in time order, and the CNN model can obtain the overall information from the local in spatial dimension. Therefore, the advantages of these two algorithms are integrated to enhance the prediction accuracy. The CNN + LSTM model designed here is the network model based on two-layer CNN and one-layer LSTM. Fig 8 reveals the algorithm flow of the CNN + LSTM model.

**Fig 8:** Algorithm flow of the CNN + LSTM model.

In Fig 8, input1 and input2 are processed by the two convolution layers, two maximum pooling layers, and a layer of the LSTM network. Then, the two LSTM network layers are connected. Finally, the feature vector of the output of the LSTM layer is mapped to a specific number by three fully connected layers, and this number is mapped between (0, 1) through the Sigmoid function to obtain the prediction results.

### Parameter setting for the model and construction of data sets

(1) Parameter setting for the model.

The two input objects are set. Take input1 as an example. The input form of data is defined as: input1 = keras. Layers. Input (shape = (16,4), name = ‘input1’), representing a 16 × 4 matrix. Then, the data enter the convolution layer, and input1 is renamed in the convolution layer. The same operation is performed on input2. Specifically, input1 is renamed as Convolution1, and input2 is renamed as Convolution2. Correspondingly, the input form of data in the convolution layer is:

Convolution1 = keras. layers. Convolution (64, 4, 1, name = ‘Convolution1’) (input1)

which indicates that the convolution layer of the first layer uses 64 convolution kernels with a length of 4 to perform convolution operation on the matrix ‘input1’. After the convolution operation, the data are processed again in the pooling layer. After the pooling layer completes the operation, the data processing of the CNN part is basically completed. Then, the data processed by the model CNN is used as the input of the LSTM model. The two LSTM network structures are connected by the concatenate function, and define the feature vector merge = keras.layers.concatenate ([lstm1, lstm2])]. Then, the merge feature vector is mapped to a particular value, and the RELU function is used as the activation function until the value is processed by the two models, to complete the classification and function prediction of DEGs.

(2) Construction of data sets

From the previous data acquisition and pre-processing, to fully train the model to achieve the real prediction of the problem, it is necessary to divide the data into the training set and the test set. The training set is used to train the model and determine parameters of the model, and the test set is used to test the performance of the model. The collected data are divided into the training set and the test set according to the ratio of 9:1, as shown in Fig 9.

**Fig 9:** Data sets of the model (a) mRNA; (b) protein.

### Environment configuration for model training

The experiment is completed in the Ubuntu16.04operating system. Besides, the model programming language uses Python 3.6, and the compilation environment uses software Anaconda. The training is completed based on the Keras framework. Keras is a Python-based deep learning framework established on TensorFlow 2.0, which can easily define and train almost all types of deep learning models.

### Verification method and evaluation methodology

(1) Confusion matrix

It is a method for classifying the predicted values, namely the matching degree between the predicted values of the model to be trained on the test set and the real values on the test set. When the predicted value is equal to the true value, the matrix attains the correct classification that is located on the diagonal of the matrix, and non-diagonal elements represent the wrong classification [30, 31].

a. Accuracy

Accuracy represents the ratio of the number of data correctly classified by the test data set to the total data in the model, and Error rate represents the ratio of the number of data incorrectly classified by the test data set to the total data in the model. The Accuracy close to 1 indicates that more data are correctly classified, and the classification effect of the model is brilliant. On the contrary, the Error rate close to 1 indicates that more data are incorrectly classified, and the model has poor classification effect [32].


$$Accuracy=\frac{TP+TN}{TP+TN+FP+FN}$$ (15)

$$Error\;rate=1‐Accuracy=\frac{FP+FN}{TP+TN+FP+FN}$$ (16)

Among Eq (15) and (16), TP denotes true positivity, TN represents true negativity, FP refers to true positivity, and FN signifies false negativity.

b. Sensitivity

Sensitivity of the model is also called the true positive rate, which is used to measure the proportion of positive samples that are correctly classified. Specificity is also called the true negative rate, which is used to measure the proportion of negative samples that are correctly classified in all sample data. The closer the Sensitivity is to 1, the better the positive samples are classified correctly. Meanwhile, the closer the Specificity is to 1, the more negative samples are classified correctly, and the classification effect of the model is better [33, 34].


$$Sensitivity=\frac{TP}{TP+FN}$$ (17)

$$Specificity=\frac{TN}{TN+FP}$$ (18)

c. ROC (Receiver Operating Characteristic) curve and AUC (Area Under roc Curve) value

The ROC curve reflects the comprehensive performance of the model based on Sensitivity and Specificity. The AUC value is a probability value, representing the area of the ROC curve, and AUC ∈ (0, 1). The larger the AUC value, the better the classification effect of the model. Otherwise, the classification effect of the model is worse. The AUC value not only considers the Accuracy of the model but also considers the Sensitivity and Specificity. Fig 10 displays the ROC curve of the model [35, 36].

**Fig 10:** ROC curve of the model.

Fig 10 displays the ROC curve of the CNN + LSTM model according to a series of different two classification methods (boundary value or decision threshold). In Fig 10, the actual positive rate (sensitivity) is the ordinate, and the false positive rate (1-specificity) is the abscissa. The area value under the ROC curve is between 1.0 and 0.5. In the case of AUC > 0.5, the AUC closer to 1 indicates a better prediction effect. The accuracy is low when AUC is 0.5 ~ 0.7, the accuracy is moderate when AUC is 0.7 ~ 0.9, and the accuracy is high when AUC is above 0.9. When AUC = 0.5, the prediction method is completely ineffective and has no prediction value. AUC < 0.5 does not conform to the actual situation, which rarely occurs in practice. The larger the area under the curve, the higher prediction accuracy. On the ROC curve, the point closest to the upper left of the coordinate diagram is the critical value with high sensitivity and specificity.

(2) Five-fold cross-validation

The cross-validation evaluates the performance of the model through the classification training of the model through the training set. The samples are divided into five subsets, among which four subsets are randomly selected as the training data set of the model, and the other one is used for verification. The harmonic mean F1-Score is used to measure the performance of the model, which can be expressed as Eq (19) [37, 38].


$$F1-\mathrm{score}=\frac{2*\mathrm{Recall}*\mathrm{Precision}}{\mathrm{Recall}+\mathrm{Precision}}$$ (19)

## Experimental results and analysis

### Analysis of lignin deposition changes in walnut fruit during endocarp hardening

From the previous experimental design, the change of lignin in the development stage of walnut endocarp is observed by phloroglucinol staining. Fig 11 displays the observation results.

**Fig 11:** Changes of lignin deposition in the thin-shell walnut during endocarp hardening.

From Fig 11, the fruit of the thin-shell walnut has basically completed the expansion and development in 50 days after full bloom, and the flesh begins to harden. In Fig 11, A denotes the transverse section of the top of the fruit, B refers to the central cross section, C represents the vertical section, and D signifies the bottom cross section. In addition, a represents the observation results in 50 days after full bloom, b denotes the observation results in 57 days after full bloom, c refers to the observation results in 78 days after full bloom, and d represents the observation results in 90 days after full bloom. In addition, Cvb represents the cardiac vascular bundle, Rld denotes the lignin deposition area, Rlu stands for the non-deposition area of lignin, Sc indicates the seed coat, Ex refers to the exocarp, Ec means the endocarp, Me signifies the mesocarp, and Sk represents the seed kernel. According to the result in 50d (A), the vascular bundle of the heart skin in the center of the fruit is first dyed red, and the top, middle and bottom of the fruit during this period are not dyed, indicating that the fruit has not begun hardening during this period. From results in 57d (B), the top, middle, and bottom of the fruit are not dyed during this period, but there are dyeing marks at the top tip, indicating that the hardening begins during this period. From 78d (C), walnut flesh is dyed, and the first place to dye is the top and bottom of the fruit, demonstrating that the first place for walnut flesh hardening is the top and bottom of the fruit. From 90d (D), the staining is further deepened and dark red, and the inner skin tissue of the hardened inner skin begins to dye, demonstrating that the inner skin is hardened horizontally from outside to inside.

### Result analysis of gene screening and functional prediction of the CNN + LSTM model

Based on the above verification and evaluation methods, the gene screening and function prediction results of DEGs of thin-shell walnuts are as follows. Fig 12 illustrates the confusion matrix of the model.

**Fig 12:** Confusion matrix of the model.

In Fig 12, the data are roughly distributed in the second and fourth quadrants, and the data in the second and fourth quadrants is much larger than that in the first and third quadrants. This result indicates that the model implemented here achieves significant screening effect on the gene screening and function prediction of DEGs of thin-shell walnuts. Moreover, the results of five-fold cross-validation of expression gene screening data are shown in Fig 13.

**Fig 13:** Results of the five-fold cross-validation of DEG screening and prediction (a: Accuracy; b: Loss).

From Fig 13(A), with the continuous progress of Epochs, the Accuracy of the established training set increases. As Epoch continues to increase, the increasing trend of Accuracy slows down, and the final Accuracy is maintained at around 92%, with the highest accuracy reaching 0.9264. In Fig 13(B), the minimum Loss value in the training set is below 0.2, and the minimum is 0.1,723 in the validation set. It shows that the model has good performance in screening and predicting DEGs. Then, the screening and prediction results of DEGs by the proposed model are compared with those of the traditional model. The results are shown in Fig 14.

**Fig 14:** Comparison of results of different algorithms.

Fig 14 indicates that the Accuracy, Precision, Recall, and F1-Score of the CNN + LSTM model implemented here are better than those of the traditional machine learning algorithms, including support vector machine (SVM), XGBoost, CNN algorithm, and random forest algorithm. In addition, compared with traditional models, the Error rate and iteration time of the CNN + LSTM model are the smallest. Moreover, the performance of the CNN + LSTM composite algorithm is better than that of the single CNN algorithm, indicating that the algorithm model reported here is more excellent in gene prediction. Fig 15 reveals the comparison of the ROC curves of CNN + LSTM model and traditional algorithms.

**Fig 15:** ROC curves of CNN + LSTM model and traditional algorithms.

Through Fig 15, compared with the other four algorithms, the CNN + LSTM model has the largest area surrounded by coordinates, and the AUC value is 0.9,796. The AUC value of the SVM algorithm is 0.8,665, and that of the random forest algorithm is 0.9,471. The AUC value of the XGBoost algorithm is 0.9,225, and that of the single CNN algorithm is 0.9,471, indicating that the CNN + LSTM model is better than four traditional algorithms.

## Conclusions

In walnut breeding and selection, the screening of differentially expressed genes and functional prediction can significantly improve the yield and quality of crops. Based on the experiment, this study establishes a neural network model to screen the genes and predict the function of walnut endocarp during hardening period. The following conclusions are drawn. The paper walnut endocarp began to harden at 57d, and the hardened inner endocarp tissue also began to stain. The results indicate that the endocarp hardened laterally from outside to inside. Besides, the highest accuracy of the CNN + LSTM model established here can attain 0.9264, and the performance of the model is better than the traditional machine learning algorithm. The AUC value in the ROC curve is 0.9796. The CNN + LSTM model is better than the traditional algorithm for the screening and function prediction of differentially expressed genes in walnut endocarp hardening stage. Although this study uses neural networks to screen and predict the function of differentially expressed genes in walnut endocarp hardening stage, some redundant data are not processed in the data collection process of model prediction. Therefore, follow-up research will deal with redundant data and employ deep learning to predict the organizational structure.

## Supporting information

S1 Data (XLSX)
